# CMaf-Inducing Protein Promotes LUAD Proliferation and Metastasis by Activating the MAPK/ERK Pathway

**DOI:** 10.1155/2022/2501846

**Published:** 2022-09-14

**Authors:** Xiao-Yan Yu, Ming Wang, Juan-Juan Qian

**Affiliations:** ^1^Respiratory Medicine, The Second Affiliated Hospital of Jiaxing University, Jiaxing, Zhejiang 314099, China; ^2^Cardiothoracic Surgery, Shulan (Hangzhou) Hospital, Hangzhou, Zhejiang 310015, China

## Abstract

**Objective:**

Previous studies have shown that cMaf-inducing protein (CMIP) promotes tumorigenesis and progression, however, the role of CMIP in lung adenocarcinoma (LUAD) and its molecular mechanism remain unclear.

**Methods:**

In this study, the Human Protein Atlas and Kaplan–Meier Plotter database were used to analyze the expression and prognostic value of CMIP in LUAD. Then, the expression levels of CMIP in LUAD tissues and cells were detected by qRT-PCR and western blot. The lentiviral vector was used to establish a stable transfected cell line, and the transfection efficiency was detected by qRT-PCR. MTT assay, colony formation assay, transwell assay, and wound healing assay were used to evaluate the function of CMIP in LUAD. In addition, the effect of CMIP on the MAPK/ERK pathway in LUAD cells was analyzed by western blot.

**Results:**

The expression level of CMIP was significantly increased in LUAD cell and tissue samples, and the high expression of CMIP was associated with overall survival (OS) and progression-free survival (PFS) in LUAD patients. In vitro experiments showed that CMIP overexpression significantly promoted the proliferation, migration, and invasion of A549 cells. CMIP knockout significantly inhibited the proliferation, migration, and invasion of H1299 cells. In addition, it was observed that the expression levels of the MAPK/ERK pathway-related proteins were significantly increased in CMIP-overexpressed A549 cells, and promoted cell proliferation, migration, and invasion, while U0126 could significantly reverse the activation of the MAPK/ERK pathway by CMIP overexpression, and inhibit the proliferation, migration, and invasion of A549 cells.

**Conclusion:**

Our study shows that CMIP, as an oncogene, is associated with poor patient prognosis, and may promote the proliferation and metastasis of LUAD by activating the MAPK/ERK pathway. Therefore, CMIP may be a new potential therapeutic target for LUAD.

## 1. Introduction

According to the latest data from GLOBOCAN in 2020, lung cancer is still the malignant tumor with the highest number of cancer-related deaths in the world, and its mortality rate accounts for about 18.0% of cancer-related deaths [1]. Nonsmall cell lung cancer (NSCLC) accounts for approximately 90% of all lung cancer types, of which adenocarcinoma (LUAD) and squamous cell carcinoma (LUSC) are the most common subtypes [2–4]. At present, radical resection, radiotherapy, and chemotherapy are the traditional methods for clinical treatment of LUAD [5, 6], but the treatment and prognosis of LUAD are poor due to the lack of precise targeting and large side effects and other adverse factors [7]. In addition, due to the high probability of postoperative recurrence and early development of metastatic propensity in LUAD patients [8], the 5-year survival rate of lung cancer patients is only 17% [9], and the 5-year relative survival rate among metastatic patients is only 5% lower[10]. Although many genes involved in LUAD tumorigenesis have been identified at this stage, only a few of them have been developed for clinical treatment. Therefore, finding potential cancer-related genes and elucidating their biological mechanisms related to tumor malignant behavior has important therapeutic significance.

Cmaf-inducing protein (CMIP) was originally discovered in the podocytes of patients with acquired idiopathic nephrotic syndrome [11]. The protein structure of CMIP consists of an N-terminal region of the pleckstrin homology domain (PH), an intermediate region containing multiple interacting docking sites (a 14-3-3 module, a PKC domain, and an SH3 domain similar to the p85, the regulatory subunit of phosphatidylinositol 3-kinase (PI3K)) and a C-terminal region containing a leucine-rich repeat (LRR) domain [12]. At present, he function of CMIP is still unclear. Previous studies have shown that intravenous injection of small interfering RNA-targeting CMIP can prevent lipopolysaccharide-induced proteinuria in rats by inhibiting the interaction between Src kinase Fyn and cytoskeletal regulator N-WASP (neural Wiskott Aldrich syndrome protein) and between adaptor proteins Nck and nephrin [11]. CMIP interacts with RelA to inhibit the degradation of I-kappaB*α* and prevent the dissociation of the NF-kappad/I-kapp*α* complex, resulting in down-regulation of NF-kB activity [13]. In addition, Kamal et al. found that CMIP has a dual effect in undifferentiated T cells, when CMIP inactivates Lck by interacting with the p85 subunit of PI3 kinase, leading to activation of the extracellular signal-regulated kinase (ERK)1/2 and P38 MAPK pathways, but when CMIP interacts with death-associated protein kinase (DAPK)-interacting protein-1 (DIP-1) and upregulates DAPK, it blocks the nuclear translocation of ERK1/2 and thus plays a key role in preventing the development of immune responses [14]. Studies have found that two isoforms of adaptor proteins of CMIP are expressed in the human brain [15, 16] and play an important role in human reading [16] and language [17]-related behavioral traits by participating in the cMaf signaling pathway. To date, little is known about CMIP in cancer. Zhang et al. showed that high expression of CMIP in gastric cancer tissue is associated with poorer clinical parameters, RFS, and OS, and CMIP works by upregulating mitogen-activated protein kinase (MAPK) Its expression plays an oncogenic role in human gastric cancer cells [18]. However, the relationship and mechanism of action of CMIP in LUAD have not been reported.

In the present study, CMIP protein expression was significantly elevated in LUAD tissue compared with normal lung tissue and correlated with poorer overall survival (OS) and progression-free survival (PFS). In addition, CMIP overexpression promoted the proliferation, migration, and invasion of lung cancer cells. Notably, CMIP overexpression activated the MAPK/ERK signaling pathways to promote LUAD development, while U0126 reversed the oncogenic effects of CMIP. It indicated that CMIP may promote the proliferation and metastasis of LUAD by activating the MAPK/ERK pathway. CMIP can be further studied as a prognostic biomarker and clinical therapeutic target for LUAD.

## 2. Materials and Methods

### 2.1. Clinical Samples

We collected a total of 20 tumor tissue samples (LUAD) and paired adjacent normal tissue (Normal) from patients diagnosed with LUAD between June 2018 and December 2020. All patients were admitted to Shulan (Hangzhou) Hospital, and all participants signed informed consent voluntarily. In this study, two pathologists diagnosed LUAD based on the pathological results, and analyzed the histological type and tumor stage of the patients according to the eighth edition of the Lung Cancer Tumor, Lymph Node, Metastasis (TNM) Staging System [19]. This study was approved by the Research Ethics Committee of Shulan (Hangzhou) Hospital (KY2022042). The study was conducted in accordance with the Declaration of Helsinki (revised 2013).

The inclusion criteria are as follows [20]: (1) Have not received chemotherapy and radiotherapy; (2) No history of any other malignant tumor within 5 years; (3) No pregnancy or breastfeeding; (4) No cardiopulmonary insufficiency and severe cardiovascular disease; (5) No severe infection and severe malnutrition.

### 2.2. Data Collection

The human protein atlas (HPA; https://www.proteinatlas.org), immunohistochemical (IHC) staining data of CMIP in normal lung tissues, and LUAD tissues were obtained. In the HPA database, protein expression was scored on four levels of undetected, low, medium, and high based on the proportion of stained cells and the intensity of staining [21].

The Kaplan–Meier Plotter database (http://www.kmplot.com) was used for survival analysis of CMIP mRNA expression in LUAD patients, including OS and PFS, to evaluate LUAD patients prognosis. The LUAD patients were divided into high-expression group and low-expression group according to the median expression value, and the “Automatically select the best cutoff” model was selected during the analysis and the threshold with the best performance was used as the cutoff value. Results are shown graphically with hazard ratios (HR) and log-rank test *P* values with 95% confidence intervals, and log-rank test *P* values of *p* < 0.05 were considered statistically significant [22].

### 2.3. Cell Culture and Transfection

Cell culture human normal lung epithelial cells (BEAS-2B) and human nonsmall cell lung cancer cell lines (A549, H460 and H1299) were purchased from American type culture collection (ATCC). The cells were cultured in DMEM or RPMI-1640 medium (GIBCO, USA) supplemented with 10% fetal bovine serum (FBS; GIBCO, USA) and 100 U/ml of penicillin streptomycin mixed antibiotics, and the cells were cultured in a humidified incubator at 37°C and 5% CO_2_.

Cell transfection CMIP siRNA plasmid (si-CMIP) and negative siRNA plasmid (siNC), empty plasmid pcDNA3.1 (Vector), and CMIP overexpression plasmid pcDNA3.1-CMIP (OE-CMIP) were designed and synthesized by Thermo Fisher Scientific. H460 and H1299 cells (1 × 10^6^ cells/mL) were seeded in 6-well plates, grouped, and transfected when the cells grew to 80%–90%. Transfected H460 cells grouped: vector group and OE-CMIP group. Transfected H1299 cells grouped: siNC group and si-CMIP group. The plasmids were transfected into H460 and H1299 cells, respectively, using Lipofectamine™ 2000 transfection reagent (11668500, Invitrogen, Thermo Fisher Scientific, Inc.) according to the manufacturer's instructions. After 6 h of transfection, the medium was changed and the cells were cultured for another 48 h. Cells are collected. Transfection efficiency was detected using qRT-PCR.

### 2.4. Quantitative Real-Time PCR Analysis (qRT-PCR)

Total RNA from cells and tissues was extracted using the TRIzol™Plus RNA Purification Kit (Invitrogen, Thermo Fisher Scientific, Inc.) according to the manufacturer's instructions, and RNA was reverse transcribed into cDNA according to the instructions of PrimeScript RTMaster Mix (Takala, Japan). Also, the concentration and purity of cDNA were checked. qRT-PCR was performed using the SYBR PremixEx Taq II kit (Takala, Japan) to detect the relative expression levels of CMIP. PCR amplification steps: 95°C for 30 s; 95°C for 5 s, 60°C for 30 s, 72°C for 45 s, 40 cycles; 72°C for 10 min. *β*-actin was used as an internal reference gene and the data were analyzed by the 2^−ΔΔ*Ct*^ method [23]. The primer sequences are shown in Table 1.

### 2.5. Cell Viability Assays

Transfected H1299 and H460 cells were seeded in 96-well plates at 5 × 10^3^ cells/well. H460 cells were treated with or without the addition of 10 *μ*M U0126 [24–26] (#9903S, Cell Signal Technology, Danvers, MA, USA). After 24 h of cell culture, 10 *µ*L of MTT (5 mg/ml) (Biyuntian, China) was added to each well, and then incubated at 37°C for 4 h. The supernatant was aspirated and 150 *μ*L of DMSO was added to each well. The absorbance of each well was measured at 570 nm using a microplate reader (Bio-Rad Laboratory, Inc.) [27]. All experiments were repeated three times.

### 2.6. Cell Colony Formation Assay

Transfected H1299 cells and H460 cells were seeded into 6-well plates at 500 cells/well, and H460 cells were treated with or without the addition of 10 *μ*M U0126. The new medium was replaced every 3 days, and after 2 weeks of culture, cells were fixed with 4% paraformaldehyde for 30 min at room temperature and stained with 0.1% crystal violet for 30 min. Photographs were taken using a light microscope (Olympus Corporation, Japan) and the number of visible colonies were manually counted. Groups of cells containing >50 cells were identified as colonies, and the number of clones in each group was counted [28]. All experiments were repeated three times.

### 2.7. Wound Healing Assay

Transfected H1299 cells and H460 cells were seeded into 6-well plates at 5 × 10^4^ cells/well, and H460 cells were treated with or without the addition of 10 *μ*M U0126. When the cells reached 90% confluency, a 20 *µ*l pipette tip was used to scratch directly on the cell monolayer and wash the cells with PBS. They were then incubated in serum-free RPMI-1640 for 24 h. Images were taken at 0 h and 24 h using a light microscope (Leica, Germany), and ImageJ software was used to quantitatively assess the wound area and calculate cell migration rates for each group [28]. All experiments were repeated three times.

### 2.8. Transwell Assay

Matrigel (364262, BD Biosciences) was coated on a 24-well transwell chamber (Costar; Corning, Inc.) at 37°C and placed in a cell incubator overnight. After suspending transfected H1299 cells and H460 cells with FBS-free medium, 100 *μ*L of cells were seeded into the upper chamber at 5 × 10^5^ cells/ml, and 500 *μ*L of RPMI-1640 containing 10% FBS was added to the lower chamber. H460 cells were treated with or without the addition of 10 *μ*M U0126. After culturing at 37°C for 24 h, cells on the underside of the membrane were fixed with 5% glutaraldehyde for 30 min at 4°C, and then stained with 0.5% crystal violet for 30 min at room temperature. Images were taken using an inverted light microscope (Leica, Germany) and invading cells in different areas were counted and analyzed using ImageJ software [29]. All experiments were repeated three times.

### 2.9. Western Blot Analysis

Transfected H1299 cells and H460 cells were seeded into 6-well plates at 1 × 10^6^ cells/well, and the cells were collected when the cells reached a certain number. Total cell and tissue proteins were extracted using RIPA lysis buffer (Beyotime, Shanghai, China) containing protease and phosphatase inhibitors. Protein concentrations were determined using the BCA protein assay kit (Beyotime). Equal amounts of protein samples (30 *μ*g/lane) were separated on 8–12% SDS–polyacrylamide gel electrophoresis (PAGE), and proteins were transferred to polyvinylidene fluoride membranes (PVDF, Immobilon-P, Millipore). Afterward, membranes were blocked with 5% skim milk or bovine serum albumin (BSA) (for phosphorylated proteins) for 1 h at room temperature. Then at 4°C with primary antibodies CMIP (PA5-65870, Invitrogen); P38 (#9212, Cell Signaling Technology); ERK (#4695, Cell Signaling Technology); p-P38 (#9215, Cell Signaling Technology); p-ERK (#4370, Cell Signaling Technology) and *β*-actin (#3700, Cell Signaling Technology) were incubated overnight. After TBST washes, the membranes were incubated with the appropriate horseradish peroxidase-conjugated secondary antibodies goat anti-rabbit IgG H&L (HRP) (ab205718, Abcam) and goat anti-mouse IgG H&L (HRP) (ab97023, Abcam) was incubated for 2 h. Images of protein bands were obtained using ECL chemiluminescent liquid (PE0010, Solebao). The target protein expression levels were calculated and normalized using Image J software.

### 2.10. Statistical Analysis

All experiments were repeated at least three times and all statistical analyses were analyzed using SPSS 26.0 software or GraphPad Prism 8.0. All data are presented as mean ± SD. Differences between multiple groups were analyzed using one-way ANOVA and Bonferroni's multiple comparison post hoc test. *P* < 0.05 was considered to be statistically significant.

## 3. Results

### 3.1. CMIP Is Upregulated in LUAD and Associated with Poor Prognosis

To determine the relationship between CMIP expression and LUAD, tissue microarray IHC according to the HPA database showed that the expression of CMIP was significantly higher in LUAD tissue than in normal lung tissue (Figure 1(a)). Similarly, CMIP protein levels were significantly elevated in LUAD tissues and cells were confirmed by qRT-PCR and Western blot analysis. It is worth noting that among the three lung cancer cell lines, CMIP expression was highest in H1299 cells and lowest in H460 cells (Figures 1(b)b–e1(e)), therefore, knockdown of CMIP in H1299 cells and overexpression of CMIP in H460 cells were selected for subsequent experimental studies. Furthermore, using Kaplan–Meier survival curves, it was found that patients with high CMIP expression in LUAD had worse OS (*P*=0.0068) and PFS (*P*=0.015) (Figure 1(f)). Therefore, these results suggest that CMIP is involved in the occurrence and development of LUAD, which is worthy of further study.

### 3.2. CMIP Overexpression Promotes H460 Cell Proliferation

In order to explore the effect of CMIP on the occurrence and development of LUAD, this study firstly transfected CMIP overexpression or knockdown plasmids into H460 and H1299 cells, respectively. qRT-PCR detection showed that in H460 cells, compared with the vector group, CMIP mRNA level in the OE-CMIP group was significantly increased (Figure 2(a)). In H1299 cells, CMIP mRNA levels were significantly decreased in the si-CMIP group compared with the siNC group (Figure 2(b)). Subsequently, the effect of CMIP expression on the viability of H460 and H1299 cells was examined by MTT. The results showed that CMIP overexpression significantly enhanced H460 cell viability compared with the vector group (Figure 2(c)), while in H1299 cells, knockdown of CMIP significantly inhibited cell viability compared with the siNC group (Figure 2(d)). In addition, the cell colony formation assay showed that CMIP overexpression significantly increased the number of H460 cell colonies compared with the vector group (Figure 2(e)). Compared with the siNC group, knockdown of CMIP significantly reduced the number of H1299 cell colonies (Figure 2(f)).

### 3.3. CMIP Overexpression Promotes H460 Cell Migration and Invasion

Subsequently, we further assessed the effect of CMIP expression on the migration and invasion of H460 and H1299 cells. The results showed that CMIP overexpression significantly promoted H460 cell migration and invasion compared with the vector group (Figures 3(a) and 3(c)), and knockdown of CMIP significantly inhibited H1299 cell migration and invasion compared with the siNC group (Figures 3(b) and 3(d)). These results indicate that high expression of CMIP promotes the occurrence and development of LUAD.

### 3.4. CMIP Overexpression Promotes Activation of MAPK/ERK Signaling Pathway

In order to explore the molecular mechanism of abnormal expression of CMIP in the occurrence and development of LUAD, this study detected the expression of the MAPK/ERK pathway-related proteins. Western blot analysis showed that knockdown of CMIP significantly reduced p-P38 and p-ERK protein expressions, and p-P38/P38 and p-ERK/ERK ratios in H1299 cells compared with the siNC group (Figures 4(a) and 4(b)). In H460 cells, CMIP overexpression significantly increased p-P38 and p-ERK protein expression, and p-P38/P38 and p-ERK/ERK ratios compared with the vector group (Figures 4(c) and 4(d)). These results suggest that the MAPK/ERK pathways may be involved in the pathogenesis of LUAD by CMIP.

### 3.5. CMIP Overexpression Promotes H460 Cell Proliferation, Migration, and Invasion by Activating the MAPK/ERK Pathway

In addition, in order to further verify whether CMIP overexpression promotes the occurrence and development of LUAD through MAPK/ERK, H460 cells were treated with 10 *μ*M U0126, and the results of MTT assay showed that compared with the OE-CMIP group, OE-CMIP + U0126 group significantly reduced the number of cells viability (Figure 5(a)). Colony formation assays also showed similar results, with U0126 intervention significantly reducing the number of H460 cell colonies compared to the OE-CMIP group (Figure 5(b)). In addition, wound healing assay and transwell analysis showed that the migration and invasion of H460 cells were significantly inhibited after U0126 intervention compared with the OE-CMIP group (Figures 5(c) and 5(d)). These results suggest that CMIP overexpression promotes the progression of LUAD by activating the MAPK/ERK pathway.

## 4. Discussion

At present, lung cancer is still one of the malignant tumors that seriously endanger human health and life [1]. With the rapid development of various omics technologies and bioinformatics, more and more genes have been identified as biomarkers for certain cancers for disease screening, diagnosis, prognosis, or further development as therapeutic targets corresponding biological reagents. Wei et al. found that EHD2 can inhibit the invasive ability of LUAD, improve patient prognosis, and can be used as a prognostic biomarker for LUAD [30]. Huang et al. showed through bioinformatics analysis and cellular experiments that high expression of GRSF1 promotes the occurrence and development of LUAD tumors and can be used as an effective prognostic biomarker for LUAD patients [31]. Previous studies have shown that CMIP, as an oncogene, promotes the progression of human gastric cancer and human glioma, and may be a potential target for the diagnosis and treatment of human glioma [18, 32]. However, so far, no studies have addressed the relationship between CMIP and LUAD. In the present study, bioinformatics analysis found that CMIP was highly expressed in LUAD tissues and correlated with poor patient prognosis. Subsequently, by detecting the expression of CMIP at the mRNA and protein levels, the results showed that the expression of CMIP in LUAD tissues and cells was significantly higher than that in the control group. These findings suggest that CMIP can serve as a prognostic biomarker for LUAD and is a new potential target worth investigating.

In order to explore the role of CMIP in LUAD and its molecular mechanism, this study found that CMIP overexpression promoted the proliferation, migration, and invasion of H460 cells through *in vitro* cell experiments, however, CMIP knockout significantly inhibited the proliferation, migration of H1299 cells, and invasive capacity, these results are consistent with Wang et al. [32]. In contrast, Zhang et al., in addition to demonstrating that CMIP knockout significantly reduced the proliferation, migration, and invasion abilities of MKN-28 gastric cancer cells, also showed that apoptosis was significantly increased after CMIP knockout by flow cytometry [18]. Based on this, the apoptotic role of CMIP in LUAD needs to be addressed in future studies.

Previous studies have shown that CMIP can directly inhibit Src kinase and cause urinary protein in mice [11]. In addition, Src homologous collagen (Shc) protein stimulates Raf through GTPase-Ras to activate the MAPK pathway, especially the ERK pathway to promote cell proliferation [33]. It has been reported that overactivation of the MAPK pathway promotes the occurrence and development of LUAD [34–36]. A previous study reported that EphA10 drives tumor progression and immune evasion by regulating the MAPK/ERK cascade in LUAD, and the MEK inhibitor U0126 significantly reversed the promoting effect of EphA10 overexpression on LUAD cells [37]. In this study, western blot experiments showed that CMIP overexpression significantly increased the expression of MAPK/ERK pathway-related proteins in H460 cells, while U0126 could significantly reversed the function of CMIP overexpression on the activation of the MAPK/ERK pathway. Therefore, CMIP may play pro-proliferation, migration and invasion effects in LUAD by activating the MAPK/ERK pathway.

To our knowledge, this study is the first to report the oncogenic role of CMIP in LUAD. Through bioinformatics analysis, clinical tissue samples and *in vitro* cell experiments, it was proved that high expression of CMIP is associated with poor prognosis of patients, and may promote the development of LUAD by activating the MAPK/ERK pathway. However, this study has some limitations. For the first time, the effect of CMIP on the malignant characteristics of LUAD by activating the MAPK/ERK pathway was not further explored in animal models by breeding CMIP knockout mice or injecting CMIP-targeting small interfering RNAs in LUAD mice. Second, epithelial-mesenchymal transition (EMT) promotes the spread of early epithelial cancer cells and is an important parameter for assessing the ability of epithelial cancer to metastasize and invade [38, 39] the degree of tumor resistance to anticancer drugs [40–42], but, which we did not explore in this study. Therefore, these issues will be addressed in future studies.

## 5. Conclusion

In conclusion, CMIP expression was significantly elevated in both LUAD cell lines and tissues, and was significantly associated with poor patient prognosis. Furthermore, CMIP promoted the proliferation and metastasis of LUAD cells by activating the MAPK/ERK pathway. Therefore, CMIP can serve as a prognostic biomarker and potential therapeutic target for LUAD.

## Figures and Tables

**Figure 1:** CMIP is upregulated in LUAD and associated with poor prognosis. (a) Immunohistochemical tissue microarray image (HPA) of CMIP protein. (b) qRT-PCR detection of CMIP mRNA levels in normal lung tissue and LUAD tissue (*n* = 20); (c) Western blot detection of CMIP protein expression in normal lung tissue and LUAD tissue (*n* = 3); (d) mRNA levels of CMIP detected by qRT-PCR in BEAS-2B, A549, H460, and H1299 cells (*n* = 3); (e) OS and PFS in LUAD patients obtained from the Kaplan–Meier plotter online database; ^*∗∗*^*P* < 0.01 vs. (Normal group or BEAS-2B group).

**Figure 2:** CMIP overexpression promotes the proliferation of H460 cells. (a/b) The mRNA levels of CMIP in H460 (a) and H1299 (b) cells after transfection were detected by qRT-PCR; (c/d) MTT assay was used to detect the difference of CMIP expression after transfection on H460 (c) and H1299 (d) Effect of cell viability. (e/f) Cell colony formation assay to assess the effect of CMIP expression on the proliferation of H460 (e) and H1299 (f) cells after transfection. ^*∗∗*^*P* < 0.01 vs. (siNC group or vector group).

**Figure 3:** CMIP overexpression promotes H460 cell migration and invasion. (a/b) The wound healing assay was used to analyze the effect of CMIP expression on the migration of H460 (a) and H1299 (b) cells after transfection. (c/d) The effect of CMIP expression on H460 (c) and H1299 (d) cell invasion after transfection was assessed using Transwell analysis. ^*∗∗*^*P* < 0.01 vs. (siNC group or vector group).

**Figure 4:** CMIP overexpression promotes activation of the MAPK/ERK pathway. (a, b) Western blot detection of P38, ERK, p-P38 and p-ERK protein expression, and the relative expression of p-P38/P38 and p-ERK/ERK in H1299 cells. (c, d) Western blot detection of P38, ERK, p-P38 and p-ERK protein expression, and the relative expression of p-P38/P38 and p-ERK/ERK in H460 cells. ^*∗∗*^*P* < 0.01 vs. (siNC group or vector group).

**Figure 5:** CMIP promotes H460 cell proliferation, migration, and invasion by activating the MAPK/ERK pathway. (a) MTT assay to detect cell viability in each group; (b) cell clone formation assay to detect the number of cell clones in each group; (c) wound healing assay to detect cell migration in each group; (d) Transwell analysis to detect cell invasion ability of each group. ^*∗*^*P* < 0.05 and ^*∗∗*^*P* < 0.01 vs. vector group, ^##^*P* < 0.01 vs. OE-CMIP group.

**Table 1:** Primers.

Gene	Sequences (5′ to 3′)
CMIP	F: AAATTCCTGAGGCGCTG
	R: CTTCAATTGCGCTGTAGGA

*β*-actin	F: TTCCTGGGCATGGAGTC
	R: CAGGTCTTTGCGGATGTC

## Data Availability

The data used to support the findings of this study are available from the corresponding author upon request.
